The article "Evaluation of the Effect of Comprehensive and Targeted Surveillance on Nosocomial Infections in Nephrology Patients" was published in 2022. Journal: J Healthc Eng.

# Evaluation of the Effect of Comprehensive and Targeted Surveillance on Nosocomial Infections in Nephrology Patients

**DOI:** 10.1155/2022/1546150

**Published:** 2022-04-29

**Authors:** Jiali Zheng, Jiuying Fei, Hongbo Li, Yan Xu

**Affiliations:** ^1^Department of Nephrology, People's Hospital of Dongxihu District, Wuhan, Hubei 430040, China; ^2^General Practitioner, Jiangjun Road Health Center, Wuhan, Hubei 430040, China; ^3^Department of Radiology, Wuhan Sixth Hospital, Affiliated Hospital of Jianghan University, Wuhan, Hubei 430015, China

## Abstract

The article summarizes the control strategy by discussing the risk factors of nosocomial infections in the nephrology department. A survey of hospitalized patients from January 2020 to December 2020 showed that there are six types of bacteria that can cause infections. The age of the patient, the risk of invasive surgery, the low use of antibiotics, and age are all independent factors that affect the risk of nosocomial infections in the patient. The more antibiotics used, the better the infection prevention effect. Among the many risk factors for patient infection, bacterial infection is the main risk factor. *Klebsiella pneumoniae* infection rate was the highest, 33.98%; *Staphylococcus aureus* infection rate was the lowest, 6.80%. Therefore, the nephrology department should focus on strengthening the prevention of *Klebsiella pneumoniae* infection, and implement early prevention and management interventions for various risk factors.

## 1. Introduction

There are many factors for nephrology patients to have an infection during hospitalization. According to the infection situation during hospitalization, combined with the patient's actual body resistance and immunity level, reasonable analysis of the possible problems of the patient's pathogen effectively control and adjust according to external and internal standards, and control and adjust patients' infection problems. It is possible to strengthen the protection and control process, control the influencing factors of exogenous infection, strengthen the internal management of the hospital environment, and improve the overall quality control layout of the hospital. With the continuous improvement of the hospital's development level, the management requirements for the hospital's information construction also continue to increase. Nowadays, hospital reliability rating has become an important standard to measure the management level of hospitals. The development and reform of hospitals are inseparable from the informatization construction of hospitals. In the years of development, the informatization construction of Chinese hospitals has made great progress and has a certain scale. But compared with foreign countries, , there is a big gap and also many problems. Nowadays, the main task of constructing informatization is to solve problems and narrow the gap, which still needs improvement in some aspects. This will be conducive for the construction of hospital information in our country, and it is also conducive for the modernization of hospital management in our country. With the advancement of modern medicine, effective management of nosocomial infections has become an important task of hospitals. According to statistics, the probability of nosocomial infections in hospitalized patients reaches 10% each year, and the economic loss is estimated to reach 20 billion yuan. In particular, nosocomial infections will also threaten the lives of other patients in the hospital. Nephrology patients have low self-immunity, the probability of infection increases significantly during hospitalization, and the patients are older and most of the patients have underlying kidney diseases and other risk factors related to infection, which lead to nephrology inpatients becoming a high-risk group of nosocomial infections.

The article "Evaluation of the Effect of Comprehensive and Targeted Surveillance on Nosocomial Infections in Nephrology Patients" was published in 2022. Journal: J Healthc Eng.

As part of hospital informatization construction, hospital monitoring is also part of medical quality management [1]. Hospital infection monitoring requires statistical analysis of a large amount of medical data, and the results are complex. In the past, manual exploration and statistical processing were used, but this search method was incomplete and extremely inefficient. It is especially important that real-time monitoring is impossible, especially for the analysis and evaluation of the rational use of antibacterial drugs in hospitals. Because there are many factors involved, it is very complicated and can only be done manually. The analysis did not give the expected results of the hospital, so hospital infection control workers are looking for a set of scientific and practical real-time monitoring software for hospital infection to solve these problems [2]. Hospital infection control includes analysis of the rational use of antibacterial drugs, hospital disinfection and hygiene monitoring, epidemic monitoring, etc. This is a professional medical problem involving multiple disciplines and experts. For the above reasons, the independent development of hospital monitoring software may be a huge and complex task. Therefore, we will continue to study the mainstream hospital sensory monitoring software in the market. The software needs to be compatible with our existing HIS, LIS, seamless connection and data integration, easy-to-use interface, and good human-computer interaction interface.

## 2. Related Work

In the comprehensive and targeted surveillance of hospital infection of patients, domestic and foreign experts have also conducted many studies. Osman MA's research addresses the existing global nephrology workforce and training capabilities. 125 UN member states responded to the entire survey, of which 121 countries responded to survey questions related to the nephrology labor force. The global density of nephrologists is 8.83 per million population (PMP), and the density of nephrologists reported in high-income countries is 28.52 PMP [3]. Saint believes that preventing medical infections remains an international priority. Although important progress has been made in preventing nosocomial infections in the past few decades, thorny issues still exist, including how to continue to improve hand hygiene and further reduce catheter-related urinary tract infections and other related complications. Perhaps, we should also be looking for “cross-innovation,” which means breakthrough discoveries can be made through research in often divergent disciplines [4]. Kim believes that confined spaces appear in medical staff spaces, outpatient spaces, and ward spaces. Since more concentrated spaces in the hospital layout will lead to higher infection rates, it is recommended to plan these spaces separately. The open space of the hospital will be planned as an independent space [5]. In order to identify bacteria in wound infections, Hao S designed an electronic nose system with a sensor array composed of 34 sensors. Eight samples of cultured *Escherichia coli*, *Staphylococcus aureus*, *Pseudomonas aeruginosa*, and their mixtures of different concentrations were detected. Using a vector machine as a classifier, no sensor array optimization is required, and the recognition rate is as high as 86.54% [6]. Most patients in the Wagener M study were proven to have secondary bacterial infections, but debridement and subsequent wound management were considered the main treatment. Common microorganisms are Enterobacteriaceae and *Enterococcus*. Antibiotics seem to play a role in the treatment of these patients, so a good antibiotic policy is strongly advocated [7]. AP C's research results indicate that liposome-encapsulated phage cocktails have great potential in the treatment of Klebsiella pneumoniae–mediated infections. Therefore, this strategy can be used as an effective method to treat wound infections caused by *Klebsiella* in individuals who do not respond to conventional antibiotic therapy [8]. These studies have provided a lot of evidence for our experiments, but due to the short research time, there are some doubts about the tested samples, so the test results need to be confirmed by everyone.

The article "Evaluation of the Effect of Comprehensive and Targeted Surveillance on Nosocomial Infections in Nephrology Patients" was published in 2022. Journal: J Healthc Eng.

## 3. System Architecture Outline Design

### 3.1. System Overview

As an important part of the construction of hospital informatization, the hospital monitoring and management information system, it includes several functional modules of subsystems such as system settings, data entry, data query, hospital statistics, suspected case detection, and infection early warning. The main functions of each subsystem are described as follows [9–11].

#### 3.1.1. System Setting Subsystem

The hospital sensor system installation includes the installation and management of various basic hospital sensor software dictionaries. The standard dictionary is expected to improve the work efficiency of operators and reduce various errors caused by manual reference. The dictionary needs to be set in detail and comprehensively. When installing and managing user rights, it can set and change user passwords, backup, retrieve, and initialize data according to user categories.

#### 3.1.2. Data Entry Subsystem

The data entry module can enter infection case data, determine the number of discharged patients, and manually enter the incidence rate. The data entry module can enter infection case data, determine the number of discharged patients, manually enter morbidity, surgical infection cases related to hospital work management, ICU patient infection monitoring data, neonatal risk monitoring data, antimicrobial drug monitoring data, needle stick injury monitoring data, environmental cleanliness monitoring data, and case report card records. This function is to facilitate the manual input of data into the computer for statistics.

#### 3.1.3. Data Query Subsystem

According to different combinations of situations, the data query module queries recorded data, infection incidence, surgical infection, patient infection, high-risk newborns, antibacterial drugs, needle stick injuries, and environmental health data from different angles.

#### 3.1.4. The Statistics Subsystem of the Hospital

Statistics of infection incidence, surgical infection, patient infection, neonatal risk, antibacterial drugs, acupuncture wounds, and environmental health data were calculated according to the departments.

#### 3.1.5. Suspected Case Search, Infection Outbreak Early Warning Subsystem

It can monitor the overall dynamics of the hospital in real time, with detection and early warning functions, to achieve early warning and reminders of the same infection case in the same department within a period of time [12].

### 3.2. Work Investigation of Hospital Infection Management Information System

After many reviews, comparisons, and analyses, combined with the actual needs of the hospital infection control workers, the hospital infection control information system used by the hospital infection control workers and the information center staff is determined. Through communication with the staff of the hospital infection department, there are 3000 cases of nosocomial infections, and the number of nosocomial infection cases per year is counted, as shown in Figure 1.

The article "Evaluation of the Effect of Comprehensive and Targeted Surveillance on Nosocomial Infections in Nephrology Patients" was published in 2022. Journal: J Healthc Eng.

It can be seen from Figure 1 that as the number of hospital beds increases, hospital infections also increase. Traditional manual search, statistics, and analysis methods are inefficient and have high error rates. Starting from the prevention and treatment of nosocomial infections, a nosocomial infection management information system was launched. This can not only solve the above problems but also pull data from different angles, draw related work plans, and meet the business needs of various related departments. The business report of the infection control system is shown in Figure 2. The use case diagram of the system function is shown in Figure 3 [13].

As the staff of the hospital information center, you need to understand the hospital infection prevention and treatment business process. This facilitates communication with business departments, satisfies their needs, and aligns the software with actual business processes. After communicating with hospital staff by visiting similar software usage conditions in other hospitals, according to the specific situation, improve the specific business process of the hospital's work. Especially, report the business process of the infection control system. If clinicians find that a patient has a nosocomial infection, they must promptly notify the nosocomial infection control department, and report the nosocomial infection to the higher-level department after the diagnosis.

The design of hospital infection science information system and the analysis of user needs are mainly realized by UML tools. It is a language used to visually model software-intensive systems. As a model language, UML allows software developers to focus on creating product models and structures. Most models are represented by diagrams. A typical modeling diagram usually consists of several blocks or boxes, contact lines and text, which are used as additional information for the model. The communication with users in the initial stage of the system is to determine the main operating modules according to the main business process.

The functional architecture of the system is represented by the basic ideas of “big to small” and “up to down” attenuation similar to structural analysis. The functional architecture of the system is an important software infrastructure. Software developers can easily visualize the functions of each module in the system through a clear system function architecture. In the development and design process, you can also perceive the function of each module according to the functional architecture diagram, and understand the relationship between the functional modules. The system function frame diagram is shown in Figure 4 [14].

The article "Evaluation of the Effect of Comprehensive and Targeted Surveillance on Nosocomial Infections in Nephrology Patients" was published in 2022. Journal: J Healthc Eng.

The state diagram of the system describes the dynamic behavior of an entity based on event reaction, and shows how the entity reacts to different events according to the current state. This enables the events and conditions of the object to reach these states, as well as the actions that occur when these states are reached. As shown in Figure 5, it is the state diagram reported by the hospital sensor card of the hospital sensor management system [15].

### 3.3. System Database Design

Basic department information table: This table is used to store the basic information of hospital departments. Most of the units and reports of the system are based on the department name. There is no correct department setting, so many units will make mistakes or produce no results. When the basic department information table is called, it is called with officeI (department number) and office (department name) as the primary keys.  Table 1 is the basic department information table [16].

Patient medical order information table: The information in the patient medical order information table is called from the HIS system through the interface. This report contains almost all the patient's medical order information. Identify and locate the patient by hospitalization ID and hospitalization number, and identify and locate the doctor's order by the doctor's order name and doctor's order number. The patient's medical order information form is mainly used for the hospital clinic to judge whether the patient is really a hospital-infected patient based on the medical advice information when reviewing the hospital's report card, and as the basis for the approval of the review. The name of the executive department and the number of the executive department are based on the statistical reports of each executive department. If it cannot be extracted from HIS, it will affect the formation of many reports. And, if the prescribed doctor cannot be extracted, the report of the doctor's statistics cannot be generated. The patient's medical order information form provides comprehensive information for auxiliary diagnosis. It has a high degree of integration, displays the original medical order in the medical order system, and provides data support for the follow-up statistical reports of the hospital sensory department from various angles. It can also more comprehensively support the inquiries, analysis, and statistics of the hospital sensor system.  Table 2 is the patient's medical order information table.

The article "Evaluation of the Effect of Comprehensive and Targeted Surveillance on Nosocomial Infections in Nephrology Patients" was published in 2022. Journal: J Healthc Eng.

### 3.4. K-Means Algorithm

The algorithm takes *k* as an input parameter and divides the object set into *k* clusters. The average value of objects in a cluster is measured by the uniformity of the cluster. These average values are considered to be the center of gravity of the cluster, or become the center of mass. We can use the squared error criterion to determine the criterion function, which is defined as follows:

(1) $$\begin{array}{c} E=\sum_{i=1}^{k}\underset{p\in Ci}{\sum }{\left|p-m_{i}\right|}^{2}. \end{array}$$

According to the different dimensions of the distance between classes, different systematic clustering methods can be carried out. There are many methods of systematic clustering, among which the most commonly used are: longest distance method, class average method, shortest distance method, intermediate distance method, variable class average method, variable method, deviation square and center gravity method, and so on. The steps of the cluster analysis system method are the same.

Define the distance between the class Gi and Gj as the distance between the two nearest samples, namely:

(2) $$\begin{array}{c} D_{ij}=\underset{Gi\in Gi\cdot Gj\in Gj}{\min}d_{ij}. \end{array}$$

Let the classes *Gp* and *Gq* be merged into a new category, denoted as *Gr*. Then, the distance between any type of *Gk* and *Gr* is:

(3) $$\begin{array}{c} Dkr=\underset{Gi\in Gi\cdot Gj\in Gj}{\min}d_{ij},\\ \min\left\{\underset{xi\in Gk\cdot xj\in Gp}{\min}d_{ij},\underset{xi\in Gk\cdot xj\in Gq}{\min}d_{ij}\right\},\\ \min\left\{D_{kp},D_{kq}\right\}. \end{array}$$

The dimension and magnitude of each attribute will be different. Therefore, some very large properties can be found in this specific calculation process, which will affect the distribution. Therefore, these quality data need to be standardized, and each attribute value is combined into a specific standard, so that the combined data have a specific set of common numerical characteristics. The method of unifying the data can be done like shown below:

(4) $$\begin{array}{c} x_{ij}=\frac{x_{ij}-{\bar{x}}_{j}}{S_{j}}, \end{array}$$

(5) $$\begin{array}{c} x_{j}=\frac{1}{n}\sum_{i=1}^{n}x_{ij}, \end{array}$$

Here, the following extreme value standardization formula can be used to calculate:

(6) $$\begin{array}{c} x_{ij}^{\prime \prime }=\frac{x_{ij}^{\prime }-x_{j\min}^{\prime }}{x_{j\max}^{\prime }-x_{j\max}^{\prime }}, \end{array}$$

(7) $$\begin{array}{c} R=\left[\begin{array}{cccc} r11 & r12 & \cdots & r1n\\ r21 & r22 & \cdots & r2n\\ \cdots & \cdots & \cdots & \cdots \\ rn1 & rn2 & \cdots & rnm \end{array}\right]. \end{array}$$

There are many commonly used methods to calculate rij, such as the distance method, geometric mean minimum method, correlation coefficient method, and angle cosine method. The Euclidean distance method is used here, and the distance coefficient is defined as *d*_*ij*_, and the *D* matrix is:

(8) $$\begin{array}{c} D=\left[\begin{array}{cccc} d11 & d12 & \cdots & d1n\\ d21 & d22 & \cdots & d2n\\ \cdots & \cdots & \cdots & \cdots \\ dn1 & dn2 & \cdots & dnm \end{array}\right], \end{array}$$

(9) $$\begin{array}{c} d_{ij}=\sqrt{\sum_{k=1}^{n}{\left(x_{ik}-x_{jk}\right)}^{2}}. \end{array}$$

Now take the first indicator as an example for data normalization:

Average is:

(10) $$\begin{array}{c} {\bar{x}}_{i}=\frac{1}{n}\sum_{i=1}^{n}x_{i1}\\ =\frac{\left(99.51+99.16+93.12+\cdots +80+78.67\right)}{23}\\ =95.41. \end{array}$$

The standard deviation is:

(11) $$\begin{array}{c} S1=\sqrt{\frac{1}{n-1}\sum_{i=1}^{n}{\left(x_{i1}-{\bar{x}}_{1}\right)}^{2}}\\ =6.47. \end{array}$$

According to (4), to get the standard value:

(12) $$\begin{array}{c} x_{11}^{\prime }=\frac{x_{11}-{\bar{x}}_{1}}{S1}\\ =\frac{\left(99.51-95.41\right)}{6.47}\\ =0.633,\\ x_{21}^{\prime }=\frac{x_{21}-{\bar{x}}_{1}}{S1}\\ =\frac{\left(99.61-95.41\right)}{6.47}\\ =0.579. \end{array}$$

According to (6), the standardized data are compressed into the closed interval [0, 1]:

(13) $$\begin{array}{c} x_{11}^{\prime \prime }=\frac{x_{11}^{\prime }-x_{\min1}^{\prime }}{x_{\max1}^{\prime }-x_{\min1}^{\prime }}\\ =\frac{\left(0.633+2.587\right)}{\left(0.709+2.587\right)}\\ =0.977,\\ x_{21}^{\prime \prime }=\frac{x_{21}^{\prime }-x_{\min1}^{\prime }}{x_{\max1}^{\prime }-x_{\min1}^{\prime }}\\ =\frac{\left(0.579+2.587\right)}{\left(0.709+2.587\right)}\\ =0.96. \end{array}$$

Setting is to establish the fuzzy similarity relationship, where the fuzzy similarity relationship between various departments is established. According to (7) and (8), the similarity relationship is calculated with the first row and second row of the matrix as examples.

(14) $$\begin{array}{c} d_{12}=\sqrt{\sum_{k=1}^{n}{\left(x_{1k}-x_{2k}\right)}^{2}},\\ \sqrt{{\left(x_{11}-x_{21}\right)}^{2}+{\left(x_{12}-x_{22}\right)}^{2}+\cdots +{\left(x_{1n}-x_{2n}\right)}^{2}}=2.072. \end{array}$$

The article "Evaluation of the Effect of Comprehensive and Targeted Surveillance on Nosocomial Infections in Nephrology Patients" was published in 2022. Journal: J Healthc Eng.

## 4. Objects and Methods of Comprehensive Research on Infection

### 4.1. The Object

Surgery departments usually include cardiothoracic surgery, general surgery, hepatobiliary surgery, neurosurgery, trauma and orthopedics, otolaryngology, urology, obstetrics and gynecology, hand and foot surgery, and burns and plastic surgery. Most of the inpatients in the hospital come from the province. The survey selected all surgical patients who were hospitalized for more than 48 hours from January 1, 2020 to December 31, 2020.

### 4.2. Exclusion Criteria

Excluding surgical patients who have not been hospitalized for more than 48 hours or who have suffered nosocomial infections before the operation shall be implemented in accordance with the regulations promulgated by the Ministry of Health. Nosocomial infections refer to infections that occur in hospitalized patients, including infections that occur during hospitalization and infections that occur in hospitals after discharge. Infections among hospital staff are also related to nosocomial infections but do not include infections before admission and infections that already existed at the time of admission.

### 4.3. Experimental Method

It collects basic information about patients undergoing surgery in the hospital, including gender, age, medical record number, department, date of admission, and basic information about surgery (days before surgery, emergency/elective schedule, anesthesia, type of surgery, operation time, etc.). The main purpose of antibiotics is whether to use antibiotics preventively, whether to use antibiotics before surgery, where and when to use antibiotics before surgery, etc. [17].

The study subjects were observed until the onset of nosocomial infections, discharge, or death. Surgery patients with nosocomial infections were included in the case group, and patients without infection during the operation were included in the control group. For surgical patients with nosocomial infections, use the nosocomial infection case questionnaire to collect more information about the patient's infection: date of infection, location of infection, etiological examination results, drug susceptibility test results, etc. According to descriptive research methods, calculate the morbidity, morbidity intensity, underreporting rate, standardized disease intensity, and other indicators of surgical patients, and calculate the distribution of hospital infection sites and departments of surgical patients. It also calculates the risk index of surgical patients. After adjusting the risk index, it calculates the morbidity and disease density of surgical patients [18].

(15) $$\begin{array}{c} \text{Incidence}=\frac{\text{Number of new hospital infections during the same period}}{\text{Number of hospitalized patients monitored during a certain period}}\times 100\%,\\ \text{Incidence rate}=\frac{\text{Number of new hospital infections during the same period}}{\text{Number of hospitalized patients monitored during a certain period}}\times 100\%,\\ \text{False negative rate}=\frac{\text{Number of underreported nosocomial infections during the same period}}{\text{The actual number of infections in a certain period}}\times 100\%,\\ \text{Incidence density}=\frac{\text{Number of new hospital infections during the same period}}{\text{Number of bed days of inpatients monitored during a certain period}}\times 100\%. \end{array}$$

The quantitative data of the study were analyzed by *t*-test or nonparametric test, case management research method was used, and the difference between the case group and the control group was analyzed by chi-square test or Fisher's exact probability method. Logistic regression analysis was performed on the research factors and the nosocomial infection factors, and the OR value of related research factors was calculated. The variables with *P* < 0.1 in the above single factor analysis were included in the multiple logistic regression model for analysis. The study uses SPSS21.0 software to analyze the relevant data. All hypothesis tests are carried out by two-sided tests, with *α* < 0.05 as the significance level for judgment.

The article "Evaluation of the Effect of Comprehensive and Targeted Surveillance on Nosocomial Infections in Nephrology Patients" was published in 2022. Journal: J Healthc Eng.

In the design stage, the design of this project has been studied and demonstrated by many experts and professors to ensure that the project design is scientific, reasonable, and feasible. Pre-survey the research objects and continuously improve the content of the questionnaire. In the project implementation stage, the investigators are trained before conducting the investigation to ensure that the investigators can clarify the purpose of the investigation, and are familiar with the content, methods, and techniques of the investigation. During the investigation, the nosocomial infection staff checked the questionnaire in time, found the wrong items and missing items, and made supplements and improvements in time. Proactively communicate with clinicians, nurses, microbiological testers, patients, or accompanying personnel in time to ensure the high efficiency of the investigation. In the data analysis stage, communicate with statistical professionals in time, find problems, and solve them in time [19]. Patients with nephropathy are mostly chronic kidney disease. Due to the long course of disease, the increased permeability of the glomerular basement membrane, and the decrease in glomerular filtration, the patient's own albumin loss is relatively large, and the patient's immune ability is low, and it is easy to be susceptible. Infection caused by pathogenic bacteria ultimately affects the clinical treatment of the primary disease, aggravates the patient's condition, and even endangers the patient's life.

The article "Evaluation of the Effect of Comprehensive and Targeted Surveillance on Nosocomial Infections in Nephrology Patients" was published in 2022. Journal: J Healthc Eng.

### 4.4. Research Situation

A total of 3804 surgical patients were investigated this time: 1741 were males, accounting for 45.7%; 2063 were females, accounting for 54.3%. There were 221 surgical patients aged 14 and under, accounting for 5.8%; 3085 surgical patients aged 15–59, accounting for 81.1%; 498 surgical patients aged 60 and above, accounting for 13.1%. The oldest is 89 years old and the youngest is 2 years old. The average age is 38.1 ± 13.9 years, of which the average age of men is 39.6 ± 13.8 years, and the average age of women is 35.1 ± 14.7 years [20]. Among all the patients investigated, 891 were in general surgery, 706 were in hepatobiliary surgery, 683 were in obstetrics and gynecology, 426 were in trauma and orthopedics, 316 were in ENT, and 247 were in neurosurgery, 210 cases of urology, 135 cases of cardiothoracic surgery, 104 cases of hand and foot surgery, and 85 cases of burn plastic surgery department.  Figure 6 shows the distribution of surgical patients in each department.

A total of 3804 surgical patients were investigated. The investigation and analysis of the use of antibacterial drugs showed that 2706 surgical patients used antibacterial drugs, and the use rate of antibacterial drugs was 71.1%. The use of antibiotics in cardiothoracic surgery, neurosurgery, urology, and foot surgery is relatively high (see Table 3 for antibiotic use in patients in various departments). Among all surgical patients who used antibacterial drugs, there were 2015 surgical patients using antibacterial drugs in combination, accounting for 74.5%; 593 surgical patients using dual antibacterial drugs, accounting for 74.5%; 593 surgical patients using dual antibacterial drugs, accounting for 21.9%; and 98 surgical patients using triple antibacterial drugs, accounting for 3.6% [21].

During the operation, there were 1880 surgical patients who used antimicrobial prophylactically, accounting for 49.4% of all surgical patients; 1037 cases of preoperative preventive medication, accounting for 55.2% of patients using prophylactic antibiotics during surgery; and 1496 cases of postoperative preventive medication, accounting for 79.6% of patients with surgical preventive medication. There were 697 patients who used antibiotics before and after surgery, accounting for 37.1% of the patients who used antibiotics preventively. The use of preventive antibiotics in neurosurgery and urology surgery is relatively high (see Table 3 for the use of preventive antibiotics in patients undergoing surgery in different departments). The average time to start medication before surgery was 36.3 hours before surgery, and the average time to medication after surgery was 4 days.

The article "Evaluation of the Effect of Comprehensive and Targeted Surveillance on Nosocomial Infections in Nephrology Patients" was published in 2022. Journal: J Healthc Eng.

This survey shows that the most commonly used antibacterial drugs are cephalosporins, which account for 40.31% of all research subjects using antibacterial drugs; followed by penicillin antibacterial drugs, accounting for 16.95% of all antibacterial drugs; aminoglycosides, accounting for 12.54%; quinolones, accounting for 11.18%; and metronidazole/tinidazolem accounting for 8.4%.  Figure 7 shows the distribution of antibacterial drugs in surgical patients [22].

Among all the surgical patients, there were 3265 elective surgery patients and 539 emergency surgery patients. There were 1685 patients undergoing general anesthesia and 2119 patients undergoing local anesthesia. There were 1694 patients with type I incision surgery, 1958 patients with type II incision surgery, and 152 patients with type III incision surgery. The average hospital stay before operation was 6.3 days, the average operation time was 118 minutes, and the average hospital stay was 14.2 days. In this survey, there were 1,050 patients who did not undergo any invasive operation, accounting for 27.6%; the number of patients who had undergone invasive operation was 2,754, accounting for 72.6%. Among them, the use rate of drainage tube accounted for 49.6%, the use rate of urinary catheter accounted for 28.7%, arteriovenous intubation accounted for 11.4%, and the remaining invasive procedures accounted for 10.3%. There were 1077 patients who had undergone more than two invasive procedures, accounting for 39.1%.

Among all surgical patients investigated, the total number of observation bed days was 32714 bed days, the number of hospital infection cases was 219, and the incidence rate of surgical patients was 5.8%; the number of infection cases was 236, and the incidence rate was 6.2%. A total of 206 cases of nosocomial infection were reported by surgical clinicians, and the underreporting rate was 12.7%.

The incidence of nosocomial infections fluctuated between 4.5% and 6.5% between January and December 2020. As shown in Figure 8, there was no statistically significant difference in the incidence of each month. The incidence density of surgical patients was 6.7‰, and the monthly incidence density fluctuated between 5.9‰ and 7.3‰. As shown in Figure 8, there was no statistically significant difference in incidence density between months. In the case group, there are 143 males, accounting for 65%; 76 females, accounting for 35%. The severity of nosocomial infections is shown in Table 4. The gender differences in nosocomial infections of surgical patients are statistically significant. Among them, the average age of men is 40.5 ± 14.1, and the average age of women is 34.9 ± 13.2 years. The incidence of nosocomial infection in each age group is shown in Table 4. The age difference of nosocomial infections among surgical patients was statistically significant [23].

The article "Evaluation of the Effect of Comprehensive and Targeted Surveillance on Nosocomial Infections in Nephrology Patients" was published in 2022. Journal: J Healthc Eng.

In the case group, nosocomial infections of patients undergoing operations in different clinical departments are mostly primary respiratory infections, but surgical infections are more common in the Department of Traumatology and Orthopedics and Hand and Foot Surgery. The structure of nosocomial infections in each case is arranged as follows: lower respiratory tract infection, surgical site infection, upper respiratory tract infection, urinary tract infection, and gastrointestinal tract, skin, and soft tissue infections. As shown in Figure 5. The lower respiratory tract is the most common site of infection, followed by the surgical site and the upper respiratory tract. Nosocomial infections of surgical patients ranked in the top 3 infections, the sum of which exceeded 80%. The incidence of lower respiratory tract infection was 2.1%, and the incidence density was 2.5%; the incidence of the surgical site was 1.7%, and the incidence density was 2.0‰; the incidence of upper respiratory tract infection was 0.9%, and the incidence density was 1.0%. The incidence of nosocomial infections in other parts of the body decreased successively.  Table 5.

First, conduct a gender and age balance test on the grouping of relevant research factors in the case group and the control group to eliminate the interference of the two confounding factors of gender and age. The results showed that there was no statistical difference between the groups; *X*^2^ test and factor Logistic regression were used to analyze the relevant factors of the case group and the control group again to investigate the risk factors. In the analysis, the first group in the grouping was used as the control group, and the other groups were compared and analyzed with the first group as the control [24].

The results showed that gender, age, preventive use of antibacterial drugs during surgery, preoperative hospital stay, surgical preparation, anesthesia method, surgical incision type, surgical duration, whether there was invasive surgery, and whether there was a disease were statistically significant (*P* < 0.05). It can be seen from Figure 9 that the incidence of nosocomial infections in male surgical patients is higher than that of female surgical patients; the incidence of nosocomial infections in surgical patients over 60 years old is higher than that of surgical patients in other age groups, and the incidence of nosocomial infections in surgical patients aged 15–59 is the lowest; the incidence of nosocomial infections in surgical patients who did not use antibacterial drugs during the operation was higher than that of patients who used preventive antibacterial drugs; hospital infections in surgical patients who were hospitalized for more than 3 days significantly exceeded those who were hospitalized for less than 3 days before surgery; the intensity of nosocomial infections in emergency surgery patients is higher than that in elective surgery patients; the nosocomial infection rate of general anesthesia patients is higher than that of local anesthesia patients; the infection intensity of nosocomial infection surgery patients in Class III surgery is significantly higher than other types of surgery patients; and the prevalence of nosocomial infections in type I patients is the lowest in surgical fracture operations. The intensity of nosocomial infections in surgical patients increases with the increase of operation time, and the operation time exceeds 6 hours, and the intensity of nosocomial infections in surgical patients is the highest; the nosocomial infection rate of patients with invasive surgery is significantly higher than that of patients with noninvasive surgery; the incidence of nosocomial infections in patients with underlying diseases is higher than that of patients without underlying diseases [25].

The article "Evaluation of the Effect of Comprehensive and Targeted Surveillance on Nosocomial Infections in Nephrology Patients" was published in 2022. Journal: J Healthc Eng.

From the multivariate logistic regression analysis, it can be seen that the OR 95% confidence interval of whether antibacterial drugs are used during the operation period is 0.957, 1.936, including 1, which may be a risk factor or a protective factor. Therefore, the classification study of whether to use antibacterial drugs during the operation is carried out, and the *X*^2^ test and logistic single factor analysis are carried out on whether to prevent the use of antibacterial drugs, the timing of medication, the course of treatment, and whether to use antibacterial drugs in combination. In the analysis, the first group was used as the control group, and the other groups were compared and analyzed with the first group as the control. The results show that if antibacterial drugs are used prophylactically during surgery, the preoperative antibacterial drug use time and the combined use time of antibacterial drugs are statistically significant; the preventive use of antibacterial drugs before surgery is not statistically significant, as shown in Figure 10. It shows that the preventive use of antibacterial drugs during surgery can reduce the intensity of nosocomial infections during surgery [26]. Preventive use of antibacterial drugs for less than 2 hours before surgery can effectively prevent nosocomial infections in surgical patients. The more antibacterial drugs used, the stronger the intensity of nosocomial infections in surgical patients.

The article "Evaluation of the Effect of Comprehensive and Targeted Surveillance on Nosocomial Infections in Nephrology Patients" was published in 2022. Journal: J Healthc Eng.

From the multivariate logistic regression, 9 risk factors of nosocomial infection in surgical patients can be obtained. For these 9 risk factors, the risk factor index of each patient is calculated. Calculation method: The basic risk factor index of surgical patients is 0. When a risk factor appears in a surgical patient, the risk factor index of the surgical patient increases by 1 point until the risk factor index of the surgical patient is calculated. Therefore, each patient's score can be divided into 0–9 points, and the corresponding risk factor index is divided into 10 levels. It can be seen from the results that surgical patients with one risk factor are the most, followed by surgical patients with two risk factors. With the increase of risk factors, the risk factor index gradually increases, the number of hospital infections also increases, and the incidence of surgical patients increases accordingly. Finally, calculate the risk index of each surgical patient to determine the average risk index, and the result is 1.7. The results of the study showed that nosocomial infection in nephrology patients was related to patient age, course of disease, length of hospital stay, diabetes mellitus, invasive procedures, high 24-hour urinary protein, and serum albumin. The older the patient is, the lower the body's autoimmunity is, and the easier it is to be invaded by pathogenic bacteria and complicated by infection; the longer the patient's disease course, the lower the renal function.

## 5. Discussion

The development of nosocomial infection work is extremely uneven, and the methods used in the nosocomial infection work carried out by major hospitals are uneven. In hospital infection surveillance research, epidemiology provides a series of research methods for it. The commonly used research methods are: cross-sectional studies, case-control studies, retrospective investigations, and prospective investigations, all of which belong to observation methods. Cross-sectional research, also known as current prevalence rate, can calculate hospital infection rate. It is the most commonly used method in descriptive epidemiological research. Most hospital infection surveillance uses this indicator. Prospective nested case-control research combines the advantages of prospective investigation. The advantage of a prospective nested case-control study is that it starts to collect patient-related data at the beginning of the study, and the selection bias and information bias are small; because the sample size required by the research is smaller than that of prospective investigations, it can save a lot of manpower, material resources, and financial resources; it can calculate the intensity of nosocomial infections; it can detect the trend of nosocomial infection epidemic or outbreak in time. It is a case-control research, and cleverly avoids its shortcomings, meets the requirements of causal research, and demonstrates the characteristics of high causal intensity. Therefore, applying the prospective nested case-control study to the nosocomial infection target surveillance study, the method is appropriate, and it will gradually receive the attention of the majority of medical staff and be widely used. With the continuous introduction of new technologies such as precision instruments and minimally invasive techniques, the damage caused by surgery is getting smaller and smaller, and the incidence of nosocomial infections caused by surgical site infections has decreased significantly. However, the use of new technologies also brings negative effects, such as increased opportunities for invasive operations and continuous updating of clinical drugs, which make bacteria continue to mutate and increase the probability of infection in nonsurgical sites. Therefore, the form of nosocomial infections is not optimistic, and targeted surveillance should be carried out in the daily work of nosocomial infection. Flexible application of epidemiological methods to nosocomial infection work, a prospective nested case-control study of inpatients. It further improves the nosocomial infection monitoring system, ensures the quality of monitoring, reduces the risk factors of nosocomial infection to a minimum, and then reduces the intensity of nosocomial infection [27].

The article "Evaluation of the Effect of Comprehensive and Targeted Surveillance on Nosocomial Infections in Nephrology Patients" was published in 2022. Journal: J Healthc Eng.

Urinary tract infection is one of the most common complications in clinical patients, and its incidence is second only to respiratory tract infection among various types of nosocomial infections. The high incidence of urinary tract infection may be caused by inappropriate indwelling catheters and frequent use of various interventional diagnostic and therapeutic measures. During the operation phase, the most prone to nosocomial infection is during the operation. The most ideal preventive antibacterial drug should be used during the entire operation. The concentration of antibacterial drugs reaches the proper concentration in the body, kills pathogenic microorganisms in the body, and achieves the purpose of preventing infection. Therefore, the use of antibacterial drugs within a certain period of time before surgery can achieve this goal. Antibacterial drugs are usually started within 30 minutes to 2 hours before surgery or during the induction of anesthesia, and are used in the operating room rather than in the ward. If the operation time exceeds 3 hours, antibacterial drugs should be added to ensure that the effective concentration of antibacterial drugs in the serum and tissues during the entire operation exceeds MIC90. Under normal circumstances, patients with type I surgery should not use antibacterial drugs. In special circumstances, antibacterial drugs should be used, and antibacterial drugs should be stopped within 24 hours after surgery. The proportion of patients with type I should not exceed 30%; patients with type II should be discontinued within 48 hours after surgery; and for type III patients should be stopped within 3–7 days. Studies have shown that there is premature medication during the operation period (average treatment time before surgery is 36.3 hours). Patients receive antibacterial treatment in the ward first, and the postoperative drug withdrawal time is later (mean medication time is 36.3 hours). The drug withdrawal time after the operation was 4 days, and the preventive effect of antibacterial drugs after the operation was not as good as that of the preoperative drugs. The use of antibacterial drugs in advance or long-term use of antibacterial drugs after surgery is not beneficial for preventing hospital infections, but it will prolong the overall medication time of patients and increase medical expenses. It may even lead to the production of drug-resistant bacteria and increase the risk of nosocomial infection [28].

The article "Evaluation of the Effect of Comprehensive and Targeted Surveillance on Nosocomial Infections in Nephrology Patients" was published in 2022. Journal: J Healthc Eng.

The results of the study showed that the pathogenic microorganisms in various parts of hospital infection in surgical patients were mainly Gram-negative bacteria, accounting for 59.0%. The second is Gram-positive bacteria, accounting for 27.7%, and fungi accounting for 8.2%, similar to previous research results. The main reason for this result is the extensive use of broad-spectrum antibacterial drugs, which inhibit the growth of most bacteria, but enable the fungi to multiply selectively. This has brought a lot of troubles in clinical practice and threatened the life safety of patients. According to the number of isolated strains, they are *Escherichia coli*, *Pseudomonas aeruginosa*, Acinetobacter baumannii, *Staphylococcus aureus*, *Klebsiella pneumoniae*, *Staphylococcus* hemolyticus, *Candida* albicans, *Enterococcus faecalis*, *Staphylococcus* epidermidis, and Intestinal *Bacillus*. The abovementioned pathogens are the more common pathogens in hospital infections, and the pathogens are selectively grown after extensive use of cephalosporin antibacterial drugs. The microbiological examination rate of hospitalized patients receiving antimicrobial treatment is not less than 30%. Conditional medical institutions should rationally select antibacterial drugs based on the results of clinical microbial specimen testing. Research shows that the microbiological examination rate of surgical patients is 38.2%, which meets the requirements. However, most surgical patients in this hospital have used antibacterial drugs before being submitted for microbiological examination, and there is an empirical phenomenon of drug use. Therefore, hospital infection professionals should increase the training of hospital infection knowledge, and correct some doctors' empirical choice of antibacterial drugs or direct use of antibacterial drugs with a wider antibacterial spectrum. According to the susceptibility test, antibiotics should be correctly selected to treat patients with nosocomial infections, so that doctors can establish the correct medication viewpoints and control the emergence of drug-resistant strains.

The article "Evaluation of the Effect of Comprehensive and Targeted Surveillance on Nosocomial Infections in Nephrology Patients" was published in 2022. Journal: J Healthc Eng.

## 6. Conclusion

There are significant differences in the incidence of infections caused by different pathogens in nephrology patients. The study of the article showed that the infection rate of *Klebsiella pneumoniae* reached 33.98%, and the infection rate of *Staphylococcus aureus* was the lowest at 6.80%. Therefore, in the Department of Nephrology, we must focus on strengthening the prevention of *Klebsiella pneumoniae* infection. There are many risk factors for infection in patients with kidney disease; among them, the older the patient, the greater the surgical invasiveness; the fewer the types of antibacterial drugs, the longer the hospital stay, and the use of glucocorticoids, the higher the risk of infection. According to the risk factors of infection, targeted prevention and clinical treatment of various infection factors are carried out to reduce the probability of infection caused by risk factors. Comprehensive monitoring and retrospective research are the foundation, which is the stage of exploring and improving hospital infection professionals to supplement experience. However, retrospective examinations are prone to deviations. Often due to the incomplete records of the original medical records, many cases of infection are undetectable, and missed diagnosis is inevitable. The survey results may not reflect the actual level of hospital infections. With the in-depth advancement of nosocomial infection control, nosocomial infection outbreak surveillance in the top three hospitals has achieved a qualitative leap from comprehensive surveillance investigations to targeted investigations in surveillance. This is essential for timely detection of nosocomial infection epidemics and outbreaks. Through the comprehensive monitoring of nosocomial infections and the continuous development of research methods, the education of the importance of reporting nosocomial infections to the majority of medical staff will be strengthened. Focus on strengthening the complete process of reporting, statistics, and analysis of infectious diseases, hospital infections, and other infections, establishing a hospital medical quality management system, real-time monitoring of hospital infections, and improving work efficiency. The ward during hospitalization should also be ventilated in time to maintain air circulation, and timely cleaning and disinfection can also minimize the spread of bacterial pathogens. At the same time, when formulating a clinical treatment plan, invasive operation treatment measures should be reduced, treatment equipment should be strictly managed to avoid bacterial accumulation, and medical staff should try to ensure aseptic operation to reduce the risk of infection of patients from the source. In addition, measures such as linking the underreporting of nosocomial infections with economic benefits have been implemented in clinics and groups. Therefore, the implementation of nosocomial infection monitoring must be based on a comprehensive and comprehensive nosocomial infection, and the data obtained will be more true and reliable. Studies have shown that about 5% of the infections of surgical patients appear after discharge from the hospital. This study only conducted research on all surgical patients during hospitalization, and did not follow-up on the discharged surgical patients. There is a certain information bias. Therefore, in future studies, discharged patients should be followed up to further understand the precise situation of the incidence of nosocomial infection. This study only involves a comprehensive tertiary hospital, and the results of the study may be different from other studies. The number of hospitals should be expanded, and the sample size should be increased to further understand the effect and feasibility of nosocomial infection surveillance of surgical patients.

The article "Evaluation of the Effect of Comprehensive and Targeted Surveillance on Nosocomial Infections in Nephrology Patients" was published in 2022. Journal: J Healthc Eng.

## Figures and Tables

**Figure 1:** The number of infections in the hospital each year.

**Figure 2:** Infection management system reporting business process and suspected case search management business process.

**Figure 3:** System Sichuan example map.

**Figure 4:** System functional architecture diagram.

**Figure 5:** The hospital sensor card system status diagram is reported.

**Figure 6:** Distribution table of surgical patients in each department.

**Figure 7:** Distribution of antibacterial drugs in surgical patients.

**Figure 8:** Intensity of nosocomial infections in each month.

**Figure 9:** Single factor analysis of factors related to nosocomial infection.

**Figure 10:** The influence of the use of antibacterial drugs during the operation on the intensity of nosocomial infections in surgical patients.

**Table 1:** Basic information of the departments of our hospital.

Serial number	Column name	Type of data	Length	Allow empty	Instruction
1	OfficeID	char	10	NOT NULL	Department number
2	Office	verchar	30		Department name
3	Officekindid	char	10		Standard department number
4	Ifdelete	bit	1	NOT NULL	Delete or not
5	Memoryid	char	10		Mnemonic
6	Standofficeid	char	10		Standard department
7	Ifcaseoffice	bit	1		Whether the case monitoring department
8	Ificrcumoffice	bit	1		Whether the environmental monitoring department
9	Ificu	bit	1		Whether ICU
10	Ifbak	bit	1	NOT NULL	Is it commonly used

**Table 2:** Patient's medical order information form.

Serial number	Column name	Type of data	Length	Allow empty	Instruction
1	ZYID	Vaechar	50	NOT NULL	Unique ID number for hospitalization
2	Patient id	Vaechar	50	NOT NULL	Hospital number
3	Visit id	Int	8		Number of hospitalizations
4	name	Vaechar	50	NOT NULL	Name
5	Flag	Int	4		Long testimony
6	Start date	Datetime	8		Open date
7	Stop date	Datetime	8		Date of suspension
8	Order days	Numeric	8		Days of medication
9	Order class	Vaechar	50		Medical order item classification name
10	Order code	Vaechar	16	NOT NULL	Order number
11	Order name	Vaechar	200	NOT NULL	Name of doctor's order
12	Order speci	Vaechar	50		Drug specifications
13	YCJL	Numeric	8		Dose
14	Dosage units	Vaechar	20		unit
15	YCSL	Numeric	8		Quantity
16	SYPC	Vaechar	50		Frequency of use
17	Usemaediway	Vaechar	50		Purpose of administration
18	Uspurpose	Vaechar	50		unit price
19	YPDJ	Numeric	8		Remark
20	Order memo	Vaechar	100		Times per day
21	MRCS	Int	1		Daily dosage
22	Qty day	Numeric	8		Total amount
23	Qty sum	Numeric	8		Executive department number
24	Execoffice code	Vaechar	20	NOT NULL	Executive department name
25	Execoffice name	Vaechar	50	NOT NULL	Prescribe doctor number
26	Bdoctor code	Vaechar	20		Name of prescribing doctor
27	Bdoctor name	Vaechar	20		Stop ordering doctor number
28	Edoctor code	Vaechar	20		Name of doctor who stopped advising
29	Edoctor name	Vaechar	20		Antibacterial drugs
30	Flag kjyw	bit	1		Antibacterial drugs

**Table 3:** The use of antibacterial drugs and preventive antibacterial drugs in surgical patients.

Department	Number of operations	Number of users	Utilization rate (%)	Preventive medication	Composition ratio (%)
Cardiothoracic surgery	134	116	86.6	94	81.4
Neurosurgery	247	203	82.2	182	89.8
Traumatology	427	341	79.9	282	82.7
General surgery	891	615	69.0	467	75.9
Hepatobiliary surgery	706	510	72.2	304	59.7
Urology	210	175	83.3	149	85.3
Hand and foot surgery	104	89	85.6	73	81.9
Five sense organs	316	164	51.9	81	49.6
Plastic surgery	85	66	77.6	21	31.5
Obstetrics and gynecology	683	427	62.5	225	52.8
Total	3804	2706	71.7	1880	69.5

The article "Evaluation of the Effect of Comprehensive and Targeted Surveillance on Nosocomial Infections in Nephrology Patients" was published in 2022. Journal: J Healthc Eng.

**Table 4:** The incidence of nosocomial infections by gender and age in the case group.

Grouping		Number of hospital infections	Incidence	Incidence density	*X* ^2^	*P* Value
Gender	Male	143	8.2	9.5		
	Female	76	3.7	4.3	7.81	0.005

Age	15–59 years old	145	4.7	5.1		
	≤14 years old	15	6.8	5.9	47.56	0.001
	≥60 years old	59	11.8	11.4		

**Table 5:** Incidence rate, incidence density, and composition ratio of nosocomial infections in various parts.

Site of infection	Number of cases	Incidence rate (%)	Incidence density (%)	Composition ratio (%)
Lower respiratory tract	81	2.1	2.5	37.0
Surgical site	65	1.7	2.0	29.7
Upper respiratory tract	34	0.9	1.0	15.5
Urinary tract	20	0.2	0.6	9.1
Gastrointestinal tract	7	0.5	0.2	3.2
Skin and soft tissue	3	0.2	0.1	1.4
Other parts	9	0.1	0.3	4.1
Total	219	6.2	6.9	100

## Data Availability

No data were used to support this study.
